This article has been retracted.

# Protective role of silymarin in a mouse model of renal Ischemia–Reperfusion injury

**DOI:** 10.1186/s13000-015-0436-4

**Published:** 2015-10-31

**Authors:** Jian Tan, Jianpeng Hu, Yonghui He, Feilun Cui

**Affiliations:** Department of Urology, Affiliated People’s Hospital of Jiangsu University, Zhenjiang, 212013 China

**Keywords:** Silymarin, Renal ischemia–reperfusion injury, Renal function

## Abstract

**Background:**

We investigated the mechanism of action of silymarin in a mouse model of renal ischemia–reperfusion injury (I/R) to ascertain its role in the treatment of I/R injury.

**Methods:**

Twenty-four C57BL/6 male mice were divided randomly into three groups: control (sham); ischemia–reperfusion (I/R); silymarin + ischemia–reperfusion (silymarin + I/R). In sham mice, an abdominal incision was made, followed by dissection of the bilateral renal pedicle, with no further cross-clamping of arteries. Silymarin + I/R mice were administered 100 mg/kg silymarin daily for 7 consecutive days before surgery, whereas I/R mice were administered (i.g.) 0.9 % saline + 0.1 % (v/v) ethanol daily for 7 consecutive days before surgery. Silymarin + I/R and I/R mice were subjected to renal ischemia to induce acute kidney injury after 45-min clamping of bilateral renal arteries. Serum levels of creatinine and blood urea nitrogen levels were measured. Periodic acid–Schiff (PAS) staining was undertaken to detect damaged renal tissue. Myeloperoxidase (MPO) activity and immunofluorescent detection of CD68 expression was undertaken for each group. Levels of inflammatory cytokines secreted by renal tissue were monitored by ELISA. Apoptosis was detected by TUNEL staining. Expression of cleaved-caspase-3, Bcl-2 and Bax was detected by western blotting.

**Results:**

Serum creatinine and blood urea nitrogen levels were elevated in silymarin + I/R and I/R groups compared with sham mice (*p* < 0.05), whereas those in the I/R group were significantly higher than in the silymarin + I/R group (*p* < 0.05). Number of damaged renal tubule cells and apoptotic cells in sham and silymarin + I/R groups was significantly lower than in I/R mice. MPO activity and secretion of inflammatory cytokines in silymarin + I/R and I/R groups was reduced (*p* < 0.05), and CD68 expression in silymarin + I/R mice was lower than in I/R mice (*p* < 0.05). Expression of cleaved-caspase-3 and Bax in the I/R group was significantly higher than in sham mice, whereas Bcl-2 expression was lower than in silymarin + I/R mice (*p* < 0.05).

**Conclusions:**

Silymarin can inhibit renal I/R injury by inhibiting release of inflammatory factors and regulating apoptosis.

## Background

Ischemia–reperfusion (I/R) is a common cause of acute kidney injury after kidney transplantation, embolism in renal arteries or cross-clamping surgery. The main cause of reperfusion injury is the large influx of calcium, oxygen free radicals and inflammatory cytokines, which cause extensive damage to tissue [1].

Silymarin is a polyphenolic flavonoid extracted from plants. It is used commonly for the treatment of drug-induced liver disease [4]. Several studies have shown that silymarin has antioxidant properties, and inhibits inflammation and apoptosis [2]. Given that kidney injury due to I/R involves oxidation, inflammation and apoptosis, we hypothesized that silymarin may have a protective role in this type of injury. Hence, we investigated the potential protective effect of silymarin in a mouse model of I/R injury.

## Methods

### Materials

Twenty-four healthy male C57BL/6 mice (6–8 weeks; 25–28 g) were purchased from the Shanghai Experimental Animal Center of Chinese Academy of Sciences (Shanghai, China). Silymarin was obtained from Sigma–Aldrich (St. Louis, MO, USA). Antibodies against caspase-3, cleaved-caspase-3, Bcl-2, Bax and glyceraldehyde 3-phosphate dehydrogenase were purchased from Cell Signaling Technology (Danvers, MA, USA). Anti-rabbit secondary antibody was obtained from Wuhan Boster (Wuhan, China). A Myeloperoxidase (MPO) Assay kit was purchased from Nanjing Jiancheng Bioengineering Institute (Nanjing, China). An enzyme-linked immunosorbent assay (ELISA) kit was obtained from eBioscience (San Diego, CA, USA).

### Animal model

Twenty-four C57BL/6 male mice were divided randomly into three groups: control (sham); ischemia–reperfusion (I/R); silymarin + ischemia–reperfusion (silymarin + I/R). The sham group underwent abdominal incision and dissection of the bilateral renal pedicle only. No further cross-clamping of arteries was undertaken on this group. Silymarin + I/R mice were administered silymarin (100 mg/kg body weight) daily for 7 consecutive days before surgery. I/R mice were administered (i.g.) physiologic (0.9 %) saline + 0.1 % (v/v) ethanol daily for 7 consecutive days before surgery. Application of experimental animals get approval of Ethics Committee.

### Preoperative preparations

After a 12-h fast, anesthesia was induced by injection of 2 % (w/v) sodium thiopental (50 mg/kg, i.p.). An incision was made into the abdominal cavity. The intestine was moved to expose the bilateral renal pedicle without damaging the renal artery. The renal artery and renal vein were occluded using a clip for 45 min, followed by reperfusion for 24 h, after which point mice were sacrificed. Blood was collected from the inferior vena cava. The left kidney was removed and fixed in 4 % (w/v) paraformaldehyde. The right kidney was placed in liquid nitrogen.

### Kidney function tests

All blood samples were left at room temperature for 30 min and centrifuged at 5000 rpm for 10 min at room temperature. Supernatants were collected, and serum concentrations of creatinine and blood urea nitrogen (BUN) measured at the People’s Hospital Affiliated with Jiangsu University.

### Pathology of kidney tissue

Serial sections (thickness, 4 μm) were washed with distilled water, incubated in 0.5–1 % (v/v) aqueous periodate for 5–10 min, and washed three times with distilled water. Sections were differentiated, followed by incubation in Schiff’s reagent for 10–30 min. After staining, sections were subjected to washing three times with sulfite, then with distilled water. Sections were counterstained with hematoxylin to identify nuclei. Grading of renal tubular necrosis was based on a points system for staining: 0 points, no damage; 1, ≤10 % tissue staining; 2, 11–25 %; 3, 26–45 %; 4, 46–75 %; 5, ≥76 %. Each sample was selected randomly. For each specimen, the mean lesion score was taken from five fields of view.

### MPO activity in kidney tissue

MPO activity in kidney tissue was measured according to manufacturer instructions. Tissue from each group was washed in 0.9 % saline and weighed to ensure equal amounts were used. Tissue was homogenized on ice in saline (1:9) and centrifuged at 12,000 rpm for 1 min at room temperature. Supernatants were added to extracts adjoining an anisidine-H_2_ reaction system, mixed and incubated for 20 min at 60 °C in a water bath. The absorbance of each tube was measured at 460 nm.

After deparaffinization and antigen retrieval, paraffin-embedded kidney sections (thickness, 2 μm) were incubated with 10 % (v/v) fetal bovine serum for 30 min, followed by incubation with rat anti-CD68 primary antibody in a moist chamber overnight at 4 °C. After washing, secondary antibodies (fluorescein isothiocyanate-conjugated rabbit anti-mouse IgG and FITC-conjugated goat anti-rat IgG) were used.

### Detection of inflammatory cytokines by ELISA

Levels of interleukin (IL)-1β, IL-6 and tumor necrosis factor (TNF)-α in kidney homogenates from each group were detected according to manufacturer instructions.

### Terminal deoxynucleotidyl transferase dUTP nick-end labeling (TUNEL)

To identify apoptotic cells in vivo, staining of paraffin-embedded sections (thickness, 6 μm) was evaluated using a TUNEL kit according to manufacturer instructions. Apoptotic cells were visualized by fluorescence microscopy and appeared yellow-green.

### Western blotting

Standard procedures for western blotting were used to monitor expression of cleaved-caspase-3, Bcl-2 and Bax. Briefly, renal tissue homogenates (50 μm) were subjected to electrophoresis on a 15 % (w/v) sodium dodecyl sulfate-polyacrylamide gel. Protein was transferred to nitrocellulose membranes, blocked with 5 % (w/v) skimmed milk overnight, and incubated with appropriate primary antibodies. Proteins were visualized and quantified using an enhanced chemiluminescence system.

### Statistical analyses

IBM SPSS Statistics, Version 19.0 (IBM, Armonk, NY, USA) was used data analyses. Data are the mean ± standard deviation. Two-way ANOVA was used to compare between multiple groups.

## Results

### Silymarin reduces serum levels of creatinine and BUN levels

Serum levels of creatinine and BUN levels in the I/R group were 22.7 ± 1.2 and 1295.7 ± 64.2 mg/L, respectively, which were significantly higher than those in sham mice (creatinine: 4.4 ± 0.2 mg/L; BUN: 291.7 ± 17.7 mg/L, *p* < 0.05). However, serum levels of creatinine and BUN levels in silymarin + I/R mice were significantly lower than those in I/R mice (creatinine: 14.0 ± 3.9 mg/L; BUN: 571.7 ± 17.0 mg/L, *p* < 0.05; Fig. 1).

**Fig. 1:** Effect of silymarin on renal tissue after renal I/R injury. Serum levels of creatinine and blood urea nitrogen (BUN) levels in the I/R group were 22.7 ± 1.2 and 1295.7 ± 64.2 mg/L, respectively, which were significantly higher than in sham mice (creatinine: 4.4 ± 0.2 mg/L; urea nitrogen: 291.7 ± 17.7 mg/L; *p* < 0.05). However, serum levels of creatinine and BUN levels in silymarin + I/R mice were significantly lower than those in I/R mice (creatinine: 14.0 ± 3.9 mg/L; BUN: 571.7 ± 17.0 mg/L; *p* < 0.05) A meamure creatinine result. B meamure urea nitrogen result

Periodic acid–Schiff (PAS) staining revealed that sham mice had normal renal tubular epithelial cells that did not change significantly. In the I/R group, the renal medullary junction showed extensive necrosis in tubular epithelial cells, cell loss and infiltration of inflammatory cells. Mice in the silymarin + I/R group showed only mild edema of tubular epithelial cells, as well as only mild necrosis and damage to renal tubules, which was reduced significantly compared with that in the I/R group (*p* < 0.05; Fig. 2). The tubular necrosis score of silymarin + I/R mice was 1.75 ± 0.16 min, which was significantly lower than that of I/R mice (4.17 ± 0.29 min; *p* < 0.05).

**Fig. 2:** Effect of silymarin on renal tissue damage and cellular architecture after renal I/R injury. Renal histologic changes in the outer medulla from mice of sham, silymarin, I/R and silymarin + I/R groups were assessed using periodic acid–Schiff (PAS) staining. Representative slides from each group (original magnification ×400) are shown. **a** Histologic damage in the outer medulla was scored by counting the percentage of tubules that displayed tubular necrosis, cast formation and tubular dilation as follows: 0, normal; 1, <10 %; 2, 10–25 %; 3, 26–50 %; 4, 51–75 %; 5, >75 %. Ten random fields of view per kidney section (×200 magnification) were used for counting. **b** Number of necrotic tubules was measured in 10 random fields per kidney section. Data are the mean ± SE (*n* = 6/group); *p < 0.05 vs. I/R.c Periodic acid–Schiff (PAS) staining image from each group

### Silymarin inhibits the inflammatory response

MPO activity in I/R mice was 52.0 ± 6.3 U/g, which was significantly higher than that in sham mice (7.6 ± 1.2 U/g; *p* < 0.05) and silymarin + I/R mice (31.8 ± 5.4 U/g, *p* < 0.05; Fig. 3).

**Fig. 3:** Effect of silymarin on MPO activity. MPO activity in the I/R group (52.0 ± 6.3 U/g) was significantly higher than that in sham mice (7.6 ± 1.2 U/g), whereas MPO activity in silymarin + I/R mice (31.8 ± 5.4 U/g) was significantly lower than in the I/R group. *p < 0.05. MPO activity in renal tissue of mouse in each group (U/g)

I/R mice had a significantly greater number of CD68-positive cells in renal tissue (12.1 ± 0.7) compared with that in silymarin + I/R mice (6.6 ± 0.8, *p* < 0.05; Fig. 4). Levels of TNF-α, IL-1β and IL-6 in the I/R group were increased significantly compared with those in sham and silymarin + I/R mice (*p* < 0.05; Table 1).

**Fig. 4:** CD68 expression in renal tissue. Number of CD68-positive cells in renal tissue from the I/R group (12.1 ± 0.7) was significantly reduced compared with that in silymarin + I/R mice (6.6 ± 0.8). *p < 0.05

**Table 1:** Levels of TNF-α, IL-1β and IL-6

Group	TNF-α (pg/mg)	IL-1β (pg/mg)	IL-6 (pg/mg)
sham	212.5 ± 5.21^c^	271.1 ± 51.37^c^	143.0 ± 31.1^c^
I/R	2114.3 ± 110.53^a^	2721.9 ± 171.22^a^	1949.0 ± 70.5^a^
I/R + silymarin	1245.7 ± 135.31^b^	1514.4 ± 36.32^b^	1009.1 ± 110.6^b^

Levels of TNF-α, IL-1β and IL-6 were increased significantly in the I/R group compared with sham and silymarin + I/R groups .c significantly reduced compared with a and b,respectively. (*p* < 0.05)

### Silymarin inhibits apoptosis

Few apoptotic cells were detected in sham mice (0.66 ± 0.3), but a significant increase was observed in I/R kidney tissue (47.67 ± 2.4, *p* < 0.05). The number of apoptotic cells in silymarin + I/R mice was significantly lower when compared with that in I/R mice (27.67 ± 3.56, *p* < 0.05; Fig. 5).

**Fig. 5:** Detection of apoptosis. Few apoptotic cells were observed in sham mice. The I/R group mice had widespread apoptosis compared with sham mice (47.67 ± 2.40, *p* < 0.05). Silymarin + I/R mice had significantly fewer apoptotic cells (27.67 ± 3.56) compared with the I/R group

Expression of Bax and cleaved-caspase-3 in sham mice was 0.80 ± 0.15 and 0.95 ± 0.13, respectively, which was significantly upregulated in I/R mice (Bax: 0.57 ± 0.09; cleaved-caspase-3: 0.38 ± 0.10; *p* < 0.05). No difference was observed for Bcl-2 expression. Expression of Bax and cleaved-caspase-3 in silymarin + I/R mice was significantly lower than that in I/R mice (Bax: 0.64 ± 0.11; cleaved-caspase-3: 0.37 ± 0.13, *p* < 0.05), whereas Bcl-2 expression was upregulated significantly compared with that in the I/R group (1.73 ± 0.32 vs. 0.13 ± 0.08, *p* < 0.05; Fig. 6).

**Fig. 6:** Protein expression. Expression of Bax and cleaved-caspase-3 in sham mice was significantly reduced compared with that in the I/R group (*p* < 0.05). A similar result was seen for silymarin + I/R mice. However, Bcl-2 expression was increased significantly (*p* < 0.05) in silymarin + I/R mice

## Discussion

Renal I/R injury is a common cause of acute kidney injury, and can lead to irreversible kidney damage, increased patient suffering and high mortality. Therefore, interventions before such injury is sustained will be beneficial. Animal models of renal I/R injury suggest that ischemic and hypoxic tissue damage is caused during restoration of renal blood flow. This damage results in the release of large amounts of mitochondrial reactive oxygen species, calcium overload and release of inflammatory cytokines that cause apoptosis and necrosis and, subsequently, kidney damage [3]. Thus, drugs that suppress inflammation, necrosis and apoptosis may have therapeutic potential.

Silymarin has antioxidant properties and is used commonly to treat drug-induced liver disease [4]. Silymarin has been shown to inhibit the NFκB signaling pathway and reduce expression of the inflammatory cytokines TNF-α, IL-1β and IL-6, resulting in inhibition of the inflammatory response [5]. Li et al. showed the protective effects of silymarin against I/R injury in the heart, liver and brain [5]. In elegant experiments using mice, Turgut et al. demonstrated that silymarin pretreatment significantly inhibited renal I/R injury, reduced malondialdehyde levels, increased expression of superoxide dismutase, and acted as an antioxidant [6]. Similarly, we have shown in mice that silymarin pretreatment can reduce necrosis of renal tubular epithelial cells, serum levels of creatinine and BUN levels, and thereby improve kidney function. Silymarin pretreatment can also significantly reduce expression of inflammatory cytokines (TNF-α, IL-1β, IL-6), suggesting that silymarin can inhibit the immune response in renal I/R and have renoprotective effects.

Apoptosis is considered one of the major mechanisms of renal I/R injury, and is triggered by certain factors in vivo*.* Therefore, inhibition of apoptosis could reduce renal I/R injury significantly. Studies have confirmed that increases in levels of TNF-α, IL-lβ and IL-6 can damage tissue by inducing apoptosis [7]. Studies have also shown that apoptosis of renal cells and the regulation of expression of Bax and Bcl-2 are closely related [8]. Bcl-2 can inhibit the generation of free radicals, overload of intracellular calcium, permeability of mitochondrial membranes, release of cytochrome c and activation of caspase-3. Bax promotes activation of cleaved-caspase-3 and apoptosis. Therefore, the ratio of Bax to Bcl-2 determines whether a cell survives or undergoes apoptosis. A recent study showed that specific knockout of p53 in renal tubular epithelial cells significantly reduces apoptotic cell death as well as subsequent renal injury and renal fibrosis [9, 10, 11]. Here, we have shown that silymarin pretreatment can significantly increase expression of Bcl-2 protein and reduce Bax expression in kidney tissue. Moreover, silymarin can inhibit cleavage of caspase-3 and thereby reduce apoptosis of renal tubular epithelial cells.

## Conclusions

Our results suggest that silymarin may have a protective role against renal I/R injury by inhibiting the inflammatory response and apoptosis. Therefore, silymarin treatment during renal I/R injury may have promising clinical applications. Nevertheless, the precise mechanism of action of silymarin requires further investigation.

## Abbreviations

ELISA: enzyme-linked immunosorbent assay
TUNEL: terminal deoxynucleotidyl transferase dUTP nick end labeling
MPO: myeloperoxidase
I/R: ischemia–reperfusion
PAS: periodic acid–schiff
